This article has been retracted.

# Zhibai Dihuang Pill Alleviates Ureaplasma urealyticum-Induced Spermatogenic Failure and Testicular Dysfunction via MAPK Signaling Pathway

**DOI:** 10.1155/2022/7174399

**Published:** 2022-02-22

**Authors:** Kai Zhang, Junhua Guo, Yong Zhu, Rui Zhang

**Affiliations:** ^1^Department of Clinical Laboratory, The Affiliated Huai'an Hospital of Xuzhou Medical University and the Second People's Hospital of Huai'an, No. 62, Huaihai Road (S.), Huaian, 223002 Jiangsu, China; ^2^Department of Andrology, Yancheng Traditional Chinese Medicine Hospital, Yancheng, Jiangsu Province 226001, China; ^3^Department of Quality Control, Jiangsu Provincial Blood Center, No. 179, Longpan Road, Xuanwu District, Nanjing, Jiangsu Province 210000, China

## Abstract

The testicles and sperm are extremely susceptible to inflammation and oxidative stress. Although Zhibai Dihuang Pill (ZDP) has been reported to treat various infertilities including male infertility induced by Ureaplasma urealyticum (UU) infection, its mechanism is still poorly understood. This study is aimed at clarifying the underlying mechanism of ZDP to protect against UU-infected male infertility. We found that UU-infected infertile rats exhibited weight loss, reduced food intake, and decreased sperm count and vitality. The administration of ZDP improved the general state and sperm motility of rats. In addition, UU infection led to spermatogenesis disorders, impaired secretory function and blood-testis barrier (BTB) of Sertoli cells, and elevated inflammation and oxidative stress. As expected, ZDP suppressed inflammation and oxidative stress to alleviate spermatogenesis disorders. Our research showed that ZDP could improve spermatogenesis disorders and testicular function primarily through the mitogen-activated protein kinase (MAPK) signaling pathway. ZDP exerts its anti-inflammatory and antioxidant effects via the MAPK signaling pathway, thus playing an important role in ameliorating spermatogenesis failure and testicular dysfunction.

## 1. Introduction

In recent years, much attention has been attached to traditional Chinese medicines (TCMs) due to their advantages in preventing and treating diseases. Zhibai Dihuang Pill (ZDP), a well-known formula containing GHB (Guan Huangbai) in TCM, which was first recorded in Jingyue quanshu in the Ming Dynasty. ZDP is one of the ancient TCMs made from *Rhizoma anemarrhenae*, *Cortex phellodendri*, *Radix rehmanniae preparata*, *Rhizoma dioscoreae*, *Fructus corni*, *Cortex moutan*, *Rhizoma alismatis*, and *Poria*. Modern pharmacological studies have found that ZDP has the effects of antioxidation, antifatigue, anti-inflammatory, antitumor, and immune-enhancing [9]. Liu et al. [10] suggest that Zhibai Dihuang Granule may regulate the complement activation and inflammatory response and enhance the ability to recognize antigens to relieve Yin-deficiency-heat (YDH) syndrome. The effects of ZDP on urokinase-type plasminogen activator (uPA) and sperm quality of infertile patients infected with Ureaplasma urealyticum (UU) were studied [5]. The results showed that UU infection caused a decrease in the uPA content of the sperm membrane and a decrease in sperm motility. ZDP may counteract the sperm membrane damaged by UU, restore the uPA content of the sperm membrane to normal, improve the fertilization ability of sperm, and effectively treat UU infectious infertility [5–9]. Zhao et al. [11] indicate that ZDP can improve diabetic nephropathy (DN) by intervening in some major metabolic pathways, such as inhibiting glucose and lipid metabolism and enhancing methylamine metabolism. ZDP has been reported to treat immune infertility, abnormal infertility of semen, infertility induced by UU, chronic prostatitis, and seminal vesiculitis combined with male infertility. However, the lack of understanding of the mechanism of ZDP greatly limits the treatment options worldwide.

Hence, our data indicated that ZDP protects UU-induced spermatogenesis disorders from inflammatory injury and oxidative damage by the MAPK signaling pathway in mice. Our findings will enrich the molecular mechanisms of ZDP as a therapeutic agent against UU-induced infertility.

## 2. Materials and Methods

### 2.1. Animals and Treatments

Adult male Sprague-Dawley (SD) rats (8-10 weeks, 300 ± 10 g) were purchased from Experimental Animal Center. All rats had access to food and water and were housed under the conditions without specific pathogens, standard humidity (55 ± 5%), and temperature (25 ± 2°C). ZDP was purchased from Foci Group Co., Ltd. (Lanzhou, China). Forty-eight male SD rats were randomly divided into six groups (*n* = 8): control group (CTL); UU infection group (UU); 643 mg/kg (low) body weight per day ZDP group (UU+L); 1286 mg/kg (medium) body weight per day ZDP group (UU+M); 2571 mg/kg (high) body weight per day ZDP group (UU+H); and 45 mg/kg body weight per day Minocycline group (UU+Mino). The doses of ZDP we selected for this research were based on a previous study [12]. And the UU group and ZDP groups (lower and medium doses) have received placebo preparations to equal the total dose of the highest dose group. General status, including body weight, hair condition, food intake, and testicular weight, was observed, and the rats were euthanized.

Animals were fasted, and water was not allowed for 12 h before modeling, and water was prohibited on the day of the experiment. Rats were anesthetized with an intraperitoneal injection of 10% chloral hydrate 4 mL/kg, iodophor was used to sterilize 2 cm above the rat external urethra, the abdominal cavity was opened, the bladder was freed, a syringe was used to exhaust the residual urine in the bladder, and then, UU standard strain solution (2.5 × 10^5^ ccu/mL, 0.6 mL/piece, animal model group) or 0.9% sodium chloride injection (0.6 mL/piece, control group) was injected, and the abdominal cavity was sutured. On the 10th day after inoculation, 5 rats were randomly selected to be sacrificed, and the culturing method was used to detect the UU of the clipped rat epididymal tissue to determine whether the modeling was successful. After the animal model is successfully established, the administration is started. The normal control group and the model group are treated with 0.9% sodium chloride injection, whose dosage is calculated according to the ratio of the animal's body weight to the surface area of the human body. The dose of the ZDP group was 2 mL/day, and that of the Minocycline group was 2 mL/day. Gavage was continued for 21 days, 2 times a day. On the 2nd day after the drug was stopped, the animals were sacrificed. Take the organization to test the following indicators.

### 2.2. Sperm Count and Mobility Assays

After the rats were sacrificed, the epididymis was collected and sperm were obtained and rinsed from the cauda epididymidis. The sperm of each animal was homogenized and diluted, respectively, with RPMI 1640 medium in a final total volume of 5 mL at 37°C for 30 min. Semen analysis was performed under a microscope with a haemocytometer to determine sperm concentration and motility. The seminal fluid was spread on clean slides and stained with Wright's staining for morphological analysis of the sperm.

### 2.3. ELISA

Serum levels of AST, ALT, IL-1*α*, IL-6, TGF-*β*, GSH/GSSG, SOD, and MDA were detected by double-antibody sandwich enzyme-linked immunosorbent assay (ELISA) kits (Elisa Biotech, Shanghai, China). To be terse, the standards and plasma samples were added to a 96-well plate previously coated with plasma serine protease inhibitor, and then, the target antibody and HRP-conjugated secondary antibody were added. HRP substrate was added after the incubation and washing. At last, the reaction was terminated by stopping solution. The optical density (OD) at 450 nm was measured within 15 min by a microtiter plate reader (FLUOstar Omega, BMG LABTECH GmbH, Germany).

### 2.4. Hematoxylin and Eosin (H&E) Staining

Testicular morphology was examined using the H&E method. The tissue slides were deparaffinized in xylene and rehydrated in gradually concentrated ethanol for 5 min. Then, they were incubated in Harris hematoxylin solution at room temperature for 10 min and rinsed in running water for 10 min and then incubated in a eosin solution at room temperature for 20 min. Finally, they were dehydrated in gradually concentrated ethanol for 3 min, cleared in xylene for 5 min, and then fixed. The nucleus was visualized in purple color, and the cytoplasm was visualized in red color. Using the light microscope with an Optilab® camera to evaluate stained tissue slides, the morphology and structure of the spermatogenic cells in the seminiferous tubules were observed and analyzed descriptively.

### 2.5. Western Blotting

RIPA buffer (FDbio Science, Shanghai, China) containing protease inhibitors was adopted in total protein extraction. BCA Protein Assay Kit (GenStar, Shanghai, China) was used for protein content quantification. A total of 20 *μ*g protein per gel lane was separated on 8%-10% polyacrylamide gels, then transferred to PVDF membranes. Membranes were blocked with 5% skim milk in Tris-buffered saline plus Tween-20 (TBST) at room temperature for 1 h and then incubated with primary antibody against ABP (Abcam, Cambridge, MA, USA, 1 : 1000), INHB (Cell Signaling Technology, Danvers, MA, USA, 1 : 1000), Tf (Abcam, Cambridge, MA, USA, 1 : 1000), occludin (Abcam, Cambridge, MA, USA, 1 : 500), claudin-3 (Proteintech, Chicago, IL, USA, 1 : 500), claudin-11 (Proteintech, Chicago, IL, USA, 1 : 500), p38 (Cell Signaling Technology, Danvers, MA, USA, 1 : 500), ERK (Abcam, Cambridge, MA, USA, 1 : 500), JUN (Abcam, Cambridge, MA, USA, 1 : 500), or GAPDH (Zhongshanjinqiao, Inc., Beijing, China, 1 : 1000) as an internal control. Then, the membranes were incubated at room temperature for 30 min, washed with TBST for 10 min three times, incubated with the corresponding secondary antibodies at room temperature for 2 h, and washed again. Western blot bands were quantified by measuring band intensity (area × OD) using the Odyssey Infrared Imaging System (LI-COR, Lincoln, NE, USA).

### 2.6. Quantitative Real-Time PCR (qRT-PCR)

qRT-PCR was used to determine the levels of ABP, INHB, Tf, occudin, claudin-3, claudin-11, IL-1*α*, IL-6, TGF-*β*, GSH/GSSG, SOD, and MDA. Primer pairs specific for these genes were designed using published rat cDNA sequences (Table 1). Following the manufacturer's instructions, total RNA was extracted by TRIzol reagent (Invitrogen, Carlsbad, USA). The SYBR Green Real-Time PCR Master Mix Kit (Toyobo, New York, USA) was used for real-time PCR amplification for the relative quantification of RNAs. Reactions were carried out in 20 *μ*L volumes containing 1 *μ*L of each primer, 1 *μ*L cDNA (500 ng), 10 *μ*L Power SYBR Green PCR Master Mix, and the rest nuclease-free water. The manufacturer's recommended cycling parameters (95°C for 10 min, 40 cycles of 95°C for 15 s, 60°C for 30 s, and 72°C for 30 s) were used for the reaction. All reactions were repeated three times. The relative expression levels were calculated after correction for the expression of *β*-actin or GAPDH as an endogenous reference using the 2^–*ΔΔ*CT^ method.

### 2.7. Data Analysis

Statistical analyses were performed using the GraphPad Prism version 5.0 software. All data were presented as the mean ± SEM. Each experiment was replicated three times independently. Statistical comparisons were performed by Student's *t*-test between two groups. Differences among groups were analyzed by one-way ANOVA by Dunnett's test. *P* < 0.05 was considered statistically significant.

## 3. Results

### 3.1. The Effects of ZDP on General Morphology of Rats

The body weight and food intake of rats were measured before and after the UU infection. No UU was detected in the control group, and rats showed obvious UU infection after modeling. UU infection caused rat weight loss, less eating, and reduced activity. As expected, ZDP treatment can lead to weight gain, increased activity, and normal eating. 45 days after treatment, the body weight and food intake decreased significantly in the UU group compared with controls, and high-dose ZDP treatment had the same effect as Minocycline, restoring body weight and food intake to normal levels (Figures 1(a) and 1(b)). To examine whether ZDP was hepatotoxic, we determined the serum ALT and AST levels. There was no statistical difference among the six groups on either ALT or AST levels (Figure 1(c)). These results indicated that ZDP can improve the general morphology of rats without hepatotoxicity.

### 3.2. The Effects of ZDP on Sperm Quality of Rats

We further explored the role of ZDP on sperm function. Compared with the control group, UU infection significantly reduced the sperm count by 80%, and the percentage of sperm in normal morphology was merely about 10%, indicating that UU infection interfered with the normal formation and maturation of sperm. However, the administration of Minocycline restored all the sperm to its initial parameters. ZDP showed a similar protective effect in UU-infected rats, with the high-dose group being the most obvious (Figures 2(a) and 2(b)). Moreover, the total number of spermatogonia and Sertoli cells in UU-infected rats was robustly decreased. ZDP consistently suppressed the reduction of Sertoli cells and androgone in a dose-dependent manner (Figures 2(c) and 2(d)). Thus, our results confirmed that ZDP could effectively improve sperm quality.

### 3.3. Correlation between ZDP Treatment and Testicular Dysfunction

The seemingly miraculous effects of ZDP might also suggest its beneficial role in maintaining testicular function. We first measured the testicular weight in each group so as to investigate the influence of ZDP on UU-infection-induced testicular dysfunction. Consistent with the above results, UU infection induced a reduction in testicular weight in rats, while the ZDP treatment group restored the testicular weight, and the high-dose group showed the best efficacy (Figure 3(a)). Histopathological examination of testicular tissues in the control group showed an intact spermatogenic tubule basement membrane, and the spermatogenic epithelium was thick. The spermatogenic cells were arranged neatly and orderly; meanwhile, spermatogonia, spermatocytes, sperm cells, and sperm could be seen from the basement membrane to the small lumen surface. A large number of sperm were arranged in a ring shape along the central lumen without any necrosis and exfoliated cells. Johnsen's score of the control group was 10. Conversely, testicular tissues in the UU infection group showed severe damage to spermatogenic tubules, spermatogenic cell shedding, and differentiation and maturation disorders. Only limited spermatogonia were seen in the seminiferous tubules, and the lumen was filled with necrotic cells.

Obvious congestion and infiltration of inflammatory factors could be seen in the interstitium. The Johnsen score of the UU infection group was 2. The histological performance of the low-dose ZDP group and the model group was similar, while the middle-dose group showed a slightly thicker spermatogenic epithelium and an increased number of spermatogenic cells. The high-dose and Minocycline groups had the most obvious improvement effect, with thicker spermatogenic epithelium, more spermatogenic cells, and spermatogenesis, and robustly reduced infiltration of inflammatory (Figures 3(b) and 3(c)).

### 3.4. Protection of ZDP against Spermatogenesis Disorders

We hypothesized that the reduced number and impaired motility of sperm resulted from defective spermatogenesis. Sertoli cells are considered to be “nurse cells,” which secrete diverse important proteins and other substances maintaining the normal development of germ cell. Androgen-binding protein (ABP), inhibin B (INHB), and transferrin (TF) have been considered to be biological markers of Sertoli cell secretory functions. We examined the expressions of ABP, INHB, and TF to evaluate the spermatogenesis. Compared with those in the control group, rats in the UU infection group exhibited decreased protein and mRNA levels of ABP, INHB, and TF, whereas high-dose ZDP significantly restored protein and mRNA levels of ABP, INHB, and TF reduced by UU infection (Figures 4(a) and 4(b)).

In addition to Sertoli cell secretory functions, the Sertoli cell tight junction (TJ) played a vital role in spermatogenesis as the major component of the blood-testis barrier (BTB) of spermatogenic epithelial. The transmembrane components of TJ formed an impermeable “seal” between adjacent Sertoli cells, thereby separating and protecting the adluminal germ cells from the systemic circulation. In order to assess the integrity of BTB, the expressions of integral membrane proteins were evaluated by western blot and qRT-PCR. UU infection resulted in decreased mRNA and protein levels of occludin, claudin-3, and claudin-11, suggesting the disruption of BTB integrity. Similarly, this deficiency was reversed by ZDP treatment, and the effect of high-dose ZDP was equivalent to Minocycline (Figures 5(a) and 5(b)). These data indicated that ZDP regulated Sertoli cell secretory functions and BTB integrity in the case of UU infection, thus protecting against spermatogenesis disorders.

### 3.5. Alleviation of Inflammation and Oxidative Stress by ZDP

Inflammation and oxidative stress have recently been suggested to play important roles in regulating supportive cell function and spermatogenesis. To assess the inflammation and oxidative stress, we first examined the inflammatory cytokines, TGF-*β*, IL-6, and IL-1*α*, in testicular tissues and serum. qRT-PCR and ELISA detection revealed that UU infection caused significantly increased expressions of TGF-*β*, IL-6, and IL-1*α* both in testicular tissues and in serum, while ZDP treatment was capable of inhibiting the secretion of these inflammatory cytokines (Figures 6(a) and 6(b)). Oxidative stress contributed to the accumulation of glutathione disulfide (GSSG), as well as a decrease in the ratio of glutathione (GSH) to GSSG. We next evaluated oxidative stress in testicular tissues and serum. We found that the administration of ZDP attenuated the increased level of malondialdehyde (MDA) and reversed the inhibition of superoxide dismutase (SOD) activity and GSH/GSSG ratio induced by UU infection (Figure 6(c)). Thus, ZDP alleviated UU infection-induced inflammation and oxidative stress in testicular tissues and serum.

### 3.6. Protection Mechanism of ZDP via the MAPK Signaling Pathway

Studies showed that IL-6 destroyed BTB by inhibiting the degradation of BTB constitutive proteins in Sertoli cells via activating the ERK-MAPK signaling pathway. Three major subfamilies of MAPK, which were known as extracellular signal-regulated protein kinase (ERK), c-Jun N-terminal kinase (JNK), and p38 MAPK, played critical roles in inflammation and oxidative stress. UU infection stimulated the phosphorylation of all three MAPK members, JNK, ERK, and p38, in the testis, compared with the control group, whereas the administration of ZDP significantly suppressed the UU infection-induced MAPK phosphorylation (Figure 7). ZDP exerted its protective effect against UU-induced spermatogenic failure and testicular dysfunction via the MAPK signaling pathway.

## 4. Discussion

Reproductive system infection is one of the main factors leading to male infertility. Lots of evidence has confirmed a high detection rate of UU pathogenic pathogens in the semen of unexplained male infertility patients, indicating the close association between UU infection and male infertility. There are several mechanisms implicated in male infertility induced by UU infection. Reichart et al. indicate that when sperm activity relies on mitochondrial oxidative phosphorylation at low pH conditions, UU fights with mitochondrial energy production and therefore impairs sperm motility and viability [13]. Wang et al. clarifies UU infection results in an increase of the microelement ratios Cu/Zn and Cd/Zn, as well as the concentrations of As and Mg in seminal fluid, which therefore leads to sperm quality decline [14]. In addition, the existence of cross-reactive antigens between UU and human sperm membrane proteins is confirmed [15]. UU-induced TNF-*α* increases sperm apoptosis and drives the lipid peroxidation of the spermatozoa plasma membrane to levels affecting the sperm fertility capacity [16]. Currently, the connection between UU infection, male infertility, and the pathogenic mechanisms is still the focus in this field. Therapeutic targets and potential drugs are in urgent need of exploration.

In the present study, we found that the number and motility of sperm in UU-infected rats decreased, and the amount and function of the Sertoli cells also declined, suggesting the spermatogenesis dysfunction. UU-infected rats tended to recover after ZDP treatment, which was involved in the inhibition of inflammatory cytokine secretion and oxidative stress imbalance. Therefore, we speculated that ZDP played a role in improving spermatogenesis disorders and testicular dysfunction by modifying inflammation and oxidative stress.

Mammalian spermatogenesis, a highly ordered and complex process of cell development and differentiation, is regulated by testicular cells (such as germ cells, Sertoli cells, Leydig cells, and peritubular cells). Sertoli cells are the only somatic cells in contact with spermatogenic cells. In view of the unique structure and function, Sertoli cells provide a suitable microenvironment for spermatogenesis and play crucial roles in regulating spermatogenesis. Endocrine and testicular paracrine/autocrine factors are known to be involved in spermatogenesis [17]. ABP has a high affinity for androgens, which can protect them from degradation via binding and transport and also has the function of controlling their bioavailability in the testis, thereby promoting the development and maturation of spermatogenic cells [18, 19]. INHB is a glycoprotein mainly produced by Sertoli cells, which can regulate the secretion of FSH through a negative feedback loop. The decrease in INHB levels is related to severely damaged testicles [20, 21]. Another biological marker of Sertoli cell secretory functions is TF, which is thought to mediate the delivery of iron. Iron is required for the normal development of germ cells during spermatogenesis [22]. Spermatogenesis also depends on the BTB, which restricts solutes from passing through the paracellular space, forming a microenvironment within the seminiferous tubules, and provides immune privileges for meiosis and meiotic cells [23, 24]. The BTB separates the seminiferous epithelium into the adluminal and basal compartments. During murine spermatogenesis, preleptotene/leptotene spermatocytes migrate from the basal to the adluminal compartment through the BTB during stages VIII-IX [22–24]. Structural analysis revealed that the principal components of the BTB, for example, claudin-3, claudin-11, occludin, and zonula occludens-1 (ZO-1), were localized at the basal and luminal sides of the preleptotene/leptotene spermatocytes during the migration stages (VIII-IX) [22]. Although we detected claudin-11, occludin, and ZO-1 throughout spermatogenesis, claudin-3 was only detected during stages VI-IX. Studies have shown that decreased claudin-3 protein in Sox8^−/−^ testes impairs the permeability of the BTB inducing male fertility in mice [25]. Our data here showed that ZDP significantly restored the ABP, INHB, and TF protein and mRNA levels reduced by UU infection. Meanwhile, the reduction in occudin, claudin-3, and claudin-11 mRNA and protein levels was reversed by ZDP treatment. These results supported the view that ZDP played a great role in improving spermatogenesis disorders induced by UU infection.

Recently, several researchers have demonstrated that UU-induced infertility and spermatogenesis disorders are related to inflammation and oxidative stress [26–28]. In view of this, to further explain the protective mechanism of ZDP on spermatogenesis, we mainly focused on inflammation and oxidative stress. TGF-*β* is a secreted cell-related polypeptide with an immunosuppressive effect on innate and adaptive immunity. TGF-*β* is capable of recognizing itself adequately, foreign or tumor-associated antigens, and inhibits the production and/or effects of proinflammatory cytokines (such as IL-1*α*, IL-6, and TNF-*α*) [29, 30]. Li et al. [31] indicate that expression levels of IL-1*α*, IL-6, and TGF-*β* are provoked in the second week after the urinary bladder is injected with UU.

In addition, the oxidative and antioxidant systems in the male reproductive system play important roles in maintaining normal physiological functions such as cell signal transduction, hormone production, sperm capacitation, acrosome reaction, and sperm motility [32]. MDA and SOD produced by excessive oxidative stress have a toxic effect on sperm cells, damage the fluidity and integrity of the sperm membrane, increase the permeability of the membrane, and reduce or even lose the sperm motility [33–35]. The free radical scavenger GSH enables the free radical scavenging reaction to continue, thereby protecting the membrane function of sperm [36, 37]. Wang et al. clarify the beneficial effect of H_2_S on testicular dysfunction mainly by anti-inflammation and antioxidation [38]. In the present study, we demonstrated that UU infection caused significantly increased expressions of TGF-*β*, IL-6, and IL-1*α* both in testicular tissues and in serum, while ZDP treatment suppressed the secretion of these inflammatory cytokines. Besides, the administration of ZDP attenuated the increased level of MDA and reversed the inhibition of SOD activity and GSH/GSSG ratio induced by UU infection. Generally, ZDP could alleviate UU infection-induced inflammation and oxidative stress in testicular tissues and serum.

Despite these findings, the exact mechanism of ZDP governing inflammation and oxidative stress remains unknown. Oxidative stress activates the MAPK signaling pathway [12], and TGF-*β* disrupts BTB integrity through the p38 MAPK pathway [39, 40]. Herein, we believed that UU infection induced oxidative stress and inflammation, with subsequent activation of the MAPK signaling pathway and impairment of Sertoli cell function, thus leading to spermatogenesis disorders. As expected, UU infection stimulated the phosphorylation of all three MAPK members, JNK, ERK, and p38, in the testis compared with the control group, whereas administration of ZDP significantly suppressed the UU infection-induced MAPK phosphorylation. Taken together, ZDP exerted its protective effect against UU-induced spermatogenic failure and testicular dysfunction via the MAPK signaling pathway.

Limitations still existed in this study. More studies in the following were needed to verify this conclusion. In addition, our current study only evaluated the ZDP formula but not the constituent since eight medicinal crude drugs, including GHB, *Rehmannia glutinosa*, *Dioscorea batatas*, *Cornus officinalis*, *Poria cocos*, *Alisma orientale*, *Paeonia moutan*, and *Anemarrhena asphodeloides* were included ZDP. In future study, we would conduct more experiments to validate our conclusion, that is, ZDP protected against UU-infected male infertility. Taken together, our research found that ZDP had the effect of protecting the testis from inflammatory and oxidative damage in rats. The MAPK signaling pathway played a crucial role in the regulation of protection mechanisms. Our findings enrich the molecular mechanisms of ZDP as a therapeutic agent against UU-induced infertility.

## Figures and Tables

**Figure 1:** The effects of ZDP on general morphology of rats: (a) relative changes in body weight in CTL, UU, UU+ZPD(L), UU+ZPD(M), UU+ZPD(H), and UU+Mino rats; (b) average daily food intake; (c) the serum ALT and AST levels were determined by ELISA. ^∗∗^*P* < 0.01 vs. the CTL group, ^#^*P* < 0.05, and ^##^*P* < 0.01 vs. the UU group. Data was shown as mean ± SD (*n* = 5).

**Figure 2:** The effects of ZDP on sperm quality of rats. (a) The number of sperm was counted by a haemocytometer. (b) The sperm morphology was performed under a microscope. (c) The numbers of Sertoli cells were counted in seminiferous tubule sections from each group. (d) The numbers of androgone were counted in seminiferous tubule sections from each group. ^∗∗^*P* < 0.01 vs. the CTL group, ^#^*P* < 0.05, and ^##^*P* < 0.01 vs. the UU group. Data was shown as mean ± SD (*n* = 5).

**Figure 3:** The correlation between ZDP treatment and testicular dysfunction: (a) relative changes in testicular weight; (b) histopathological examination of the rat's testicular tissues with H&E stain. Scale bar, 100 *μ*m; (c) the statistics of H&E histopathological classification. ^∗∗^*P* < 0.01, ^∗∗∗^*P* < 0.001 vs. the CTL group, ^#^*P* < 0.05, and ^##^*P* < 0.01 vs. the UU group. Data was shown as mean ± SD (*n* = 5).

**Figure 4:** The influence of ZDP on Sertoli cell secretory function. (a) The levels of ABP, INHB, and TF were determined by qRT-PCR. (b) The levels of ABP, INHB, and TF were determined by western blot assay. ∗∗*P* < 0.01 vs. the CTL group, ^#^*P* < 0.05, and ^##^*P* < 0.01 vs. the UU group. Data was shown as mean ± SD (*n* = 5).

**Figure 5:** The influence of ZDP on Sertoli cell tight junction. (a) The levels of Occludin, claudin-3 and claudin-11 were determined by qRT-PCR. (b) The levels of Occludin, claudin-3, and claudin-11 were determined by western blot assay. ^∗∗^*P* < 0.01 vs. the CTL group, ^#^*P* < 0.05, and ^##^*P* < 0.01 vs. the UU group. Data was shown as mean ± SD (*n* = 5).

**Figure 6:** Alleviation of inflammation and oxidative stress by ZDP. (a) The levels of IL-1*α*, IL-6, and TGF-*β* in testicular tissues were determined by qRT-PCR. (b) The levels of IL-1*α*, IL-6, and TGF-*β* in serum were determined by ELISA. (c) The levels of GSH/GSSG ratio, SOD, and MDA in testicular tissues and serum were determined by qRT-PCR and ELISA. ^∗∗^*P* < 0.01 vs. the CTL group, ^#^*P* < 0.05, and ^##^*P* < 0.01 vs. the UU group. Data was shown as mean ± SD (*n* = 5).

**Figure 7:** Protection mechanism of ZDP via the MAPK signaling pathway. The levels of p38, p-p38, Erk, p-Erk, JNK, and p-JNK were determined by western blot assay. ^∗∗^*P* < 0.01 vs. the CTL group, ^#^*P* < 0.05, and ^##^*P* < 0.01 vs. the UU group. Data was shown as mean ± SD (*n* = 5).

**Table 1:** Primer sequences for qRT-PCR.

Gene	Primer sequences (5′-3′)
IL-1*α*	Forward: GACCATCTGTCTCTGAATCAG Reverse: CGATGAGTAGGCATACATGTC
IL-6	Forward: CTAGGAAGAACTGGCAATATG Reverse: AAACCATCTGGCTAGGTAAGA
TGF-*β*	Forward: CCGCAACAACGCAATCTAT Reverse: GAAAGCCCTGTATTCCGTCTC
ABP	Forward: TGCCCTGGATGGCTGTAT Reverse: TGTCCCTGTCCCAAGAGTAAG
INHB	Forward: CTCTGCTGCTCCTTTTG Reverse: TGGTGGCTGCGTATGTG
Tf	Forward: GCAGGATGAAGGGAGGACAC Reverse: GCGATCTGTCAGAGCACCTC
Occudin	Forward: CAGCAGCAGTGGTAACTTGG Reverse: CAGCAGCAGTGGTAACTTGG
Claudin-3	Forward: GCCAAAGCCAAGATCCTCTA Reverse: GTAGTCCTTGCGGTCGTAGG
Claudin-11	Forward: CTGGTGGACATCCTCATCCT Reverse: AGCTAGAGCCCGCAGTGTAG
GAPDH	Forward: GGTGCTGAGTATGTCGTGGAG T Reverse: CAG TCT TCT GAG TGG CAG TGA T

## Data Availability

All data generated or analyzed during this study are included in this published article.
